# Podocyte Expression of Membrane Transporters Involved in Puromycin Aminonucleoside-Mediated Injury

**DOI:** 10.1371/journal.pone.0066159

**Published:** 2013-06-20

**Authors:** Cristina Zennaro, Maria Pia Rastaldi, Lorella Pascolo, Marco Stebel, Elisa Trevisan, Mary Artero, Claudio Tiribelli, Vittorio Di Maso, Michele Carraro

**Affiliations:** 1 Department of Medical, Surgery and Health Sciences, Università degli Studi di Trieste, Trieste, Italy; 2 Renal Research Laboratory, Fondazione IRCCS Ca’ Granda Ospedale Maggiore Policlinico & Fondazione D’Amico per la Ricerca sulle Malattie Renali, Milano, Italy; 3 Department of Life Sciences, Università degli Studi di Trieste, Trieste, Italy; 4 Azienda Ospedaliero-Universitaria Ospedali di Riuniti di Trieste, Trieste, Italy; 5 Liver Research Center, AREA Science Park, Trieste, Italy; 6 IRCCS Burlo Garofolo Istituto per la Cura a Carattere Scientifico Materno Infantile, Trieste, Italy; University of Cambridge, United Kingdom

## Abstract

Several complex mechanisms contribute to the maintenance of the intricate ramified morphology of glomerular podocytes and to interactions with neighboring cells and the underlying basement membrane. Recently, components of small molecule transporter families have been found in the podocyte membrane, but expression and function of membrane transporters in podocytes is largely unexplored. To investigate this complex field of investigation, we used two molecules which are known substrates of membrane transporters, namely Penicillin G and Puromycin Aminonucleoside (PA).

We observed that Penicillin G pre-administration prevented both *in vitro* and *in vivo* podocyte damage caused by PA, suggesting the engagement of the same membrane transporters by the two molecules. Indeed, we found that podocytes express a series of transporters which are known to be used by Penicillin G, such as members of the Organic Anion Transporter Polypeptides (OATP/Oatp) family of influx transporters, and P-glycoprotein, a member of the MultiDrug Resistance (MDR) efflux transporter family.

Expression of OATP/Oatp transporters was modified by PA treatment. Similarly, *in vitro* PA treatment increased mRNA and protein expression of P-glycoprotein, as well as its activity, confirming the engagement of the molecule upon PA administration.

In summary, we have characterized some of the small molecule transporters present at the podocyte membrane, focusing on those used by PA to enter and exit the cell. Further investigation will be needed to understand precisely the role of these transporter families in maintaining podocyte homeostasis and in the pathogenesis of podocyte injury.

## Introduction

Pathology of the podocyte underlies several glomerular diseases, the most severe being focal segmental glomerulosclerosis, which is clinically characterized by heavy proteinuria or nephrotic syndrome and frequently progresses to renal insufficiency. The cellular mechanisms resulting in proteinuria are not completely understood, and thus the description of pathways leading to podocyte damage and repair are relevant to the identification of novel treatment strategies.

The membrane transport system, known as a major transmembrane component involved in the movement of ions, small molecules, and drugs, has been extensively studied in some organs and cellular systems, such as the intestine, the liver, and the blood-brain barrier. In the kidney, several members of the main membrane transporter families have been described in the renal tubule in the context of ion and drug transport [1]. Recently, two transporters with broad specificity for small molecules have been identified in mouse podocytes in relation to drug clearance [2], [3].

Podocytes are highly differentiated cells with a complex ramified structure, the maintenance of which requires coordinated trafficking from the extracellular to the intracellular compartment, similar to that operating in other highly ramified cells, such as neurons [4]. Small molecule transporters constitutively expressed in the podocyte contribute to maintain the cellular structure and barrier function, possibly by interacting with endogenous substrates and metabolites; and they could also be involved in the uptake and efflux of drugs in these cells.

A better understanding of transport mechanisms in podocytes is needed to explain in part some functions of these cells and to conform to the recently issued FDA draft guidance which includes the recommendation to increase knowledge about drug transport and metabolism (www.fda.gov/downloads/Drugs/GuidanceComplianceRegulatoryInformation/Guidances/UCM292362.pdf).

With this background, we performed experiments using Penicillin G, a well-known beta-lactam antibiotic, which is the substrate of several transporter families that have been fully characterized in other cellular models [5]. The antibiotic was used in the context of podocyte injury by puromycin aminonucleoside (PA), a small molecule that uses membrane transporters to enter the cell [6], and induces podocyte damage which mimics lesions of minimal change disease or focal segmental glomerulosclerosis, with appearance of severe proteinuria when injected in rats [7].

We reasoned that if Penicillin G engaged transporters at the podocyte surface, the entrance and the subsequent activity of PA would be blocked, providing evidence that the two molecules use the same membrane transporter families in podocytes.

## Materials and Methods

### Animals and experimental design

Young male Sprague-Dawley rats (n  = 30) weighing 230–250 g housed at the University of Trieste (Italy) animal facility were randomly divided into three control groups and three experimental groups (5 animals per each group, see Table 1). The rats were housed two or three per cage in an air-conditioned, light-controlled environment, and all animals had unrestricted access to food and water.

**Table 1:** Experimental animal groups.

Group	Treatment
Control 1 - saline	Saline solution
Control 2 - PEN 12,500	Penicillin G 12,500 Units + saline
Control 3 - PEN 15,000	Penicillin G 15,000 Units + saline
Experimental 1 - PA	Puromycin aminonucleoside (5 mg/100 g body weight)
Experimental 2 - PEN (12,500) + PA	Penicillin G 12,500 Unit + PA (5 mg/100 g body weight)
Experimental 3 - PEN (15,000) + PA	Penicillin G 15,000 Unit + PA (5 mg/100 g body weight)

A committee of the Italian Health Ministry approved the experimental protocol (prot. n 166-date: April, 8, 2005), in compliance with Italian regulation (D.L.vo 116/92). General anaesthesia was provided with an IP injection of 2 ml Avertin 2% and 100 ul Xilazine 2%. Local anaesthesia was provided with 100 ul of Lidocaine 2% in the site of incision and all efforts were made to minimize suffering.

In the experimental groups rats received a single intravenous injection (5 mg/100 g body weight) of puromycin aminonucleoside (PA) (Sigma) in the femoral vein, whereas rats in the control groups were treated with the same volume (1 ml) of saline. Pre-treatment with Penicillin G (Penicillin G sodium salt, Sigma), at dosages of 12,500 IU or 15,000 IU was performed 10 minutes before the injection of PA or saline in the same femoral vein.

A 24h urine collection was obtained on day –1 before PA injection, then on day 5 and 10.

On day 10 the animals were sacrificed, and a blood sample was collected for creatinine and serum albumin analysis. One kidney was immediately excised to isolate glomeruli for the albumin permeability tests (Palb), and the other kidney was used for histological analyses. Creatinine and serum albumin were determined by an autoanalyzer technique (Hitachi 717, Tokyo), and proteinuria was assessed by the Comassie Brillant Blue assay.

### Glomerular morphometric analysis

Kidney tissue was fixed in formalin and embedded in paraffin using standard techniques. 4 um-thick sections were deparaffinized, hydrated and stained with periodic acid-Schiff (PAS). Twenty glomeruli per animal were analyzed. Digital images were taken using an upright microscope (Olympus Italia, Segrate, Milan, Italy) equipped with a digital camera. The mean area of each glomerulus was measured by manually tracing the glomerular outline on 200X acquired images, and measured off-line by a video-based image analysis program (Sigma Scan Pro, Jandel Scientific Software).

### The convective glomerular albumin permeability assay (Palb)

The method for measuring glomerular albumin permeability, adapted from the original description by Savin [8], allows the study of the glomerular response to various mediators in the absence of systemic humoral, hemodynamic, or rheologic forces [9], and has been applied extensively by our group to analyze glomerular damage [10], [11], [12].

Glomeruli were isolated by sieving in BSA solution; during the sieving process, they are stripped of Bowman’s capsule, tubules, and associated blood vessels. In this work, two sets of experiments were performed, one comprising isolated glomeruli from control and experimental rats, and the other conducted on glomeruli isolated from untreated, healthy male Sprague Dawley rats. Glomeruli from experimental rats underwent directly Palb determination. Glomeruli from untreated animals were instead incubated with PA (0.6 ug/ml to 10.0 ug/ml) or saline for 10 minutes at 37°C. In this set of experiments Penicillin G (50 IU/ml to 700 IU/ml) was added to the incubation medium 10 min before or 10 min after PA incubation, and glomeruli were carefully washed to avoid any possible extracellular interaction between the two drugs. Penicillin G alone at the same concentration was used as a control.

### Isolated glomeruli adhesion assay

Isolated glomeruli from healthy young male Sprague Dawley rats were centrifuged at 800 rpm for 2 minutes for fragment elimination. The pellet was resuspended in medium and plated on type IV collagen-coated 24 multi-well plastic plates (100 glomeruli/well). After pre-incubation for 30 minutes with Penicillin G 500 IU/ml or 700 IU/ml, the glomeruli were carefully washed and treated with PA (10, 5 and 2.5 ug/ml) or an equal volume of incubation medium as a control. After 5 days the plates were washed to eliminate unattached glomeruli and analyzed by an inverted microscope (Leica Microsystem GmbH, Germany) to evaluate morphology and number. Three independent experiments for each concentration of Penicillin G and PA were performed.

### Podocyte cultures

We used a human immortalized cell line, following the procedure originally described by Doublier at al. [13], with minor modifications. Differentiated podocytes were cultured in Dulbecco’s modified Eagle’s high glucose medium (DMEM) containing 10% fetal bovine serum (FBS-Euroclone Ltd, Wetherby West Yorkshire, UK).

For primary podocyte cultures, glomeruli from healthy young male Sprague Dawley rats were isolated by sieving, then seeded in culture flasks pre-coated with collagen IV (Sigma Aldrich) in medium containing Dulbecco’s modified Eagle/F12 medium (DMEM/F12) supplemented with 10% FBS, 5 ug/ml transferrin, 10^−7^M hydrocortisone, 5 ng/ml sodium selenite, 0.12 U/ml insulin, 100 ug/ml Penicillin, 100 µg/ml streptomycin, 2 mM L-glutamine (Sigma-Aldrich). After four days first passage podocytes were separated from glomeruli by an additional sieving through a 40 um mesh (BD Falcon). Cell characterization was performed by immunofluorescence and PCR amplification, using podocyte markers (nephrin, podocin, WT-1).

### Penicillin fluorescence in live cells

For internalization studies we used a fluorescent Penicillin (Bocillin 650/665 Penicillin, Life Technologies Italia, Monza, Italy) to determine if the antibiotic is transported into the podocyte cytoplasm. Bocillin TM 650-655 Penicillin is a synthesized compound from Penicillin V and the Bodipy 650/655 dye.

Human podocytes were seeded on thermanox coverslips (Nunc, VWR International, Milan, Italy) in the absence of conventional antibiotic treatment. Cells were washed in HBSS buffer (Hepes 10 mmol/L, NaCl 150 mmol/L, KCl 5 mmol/L, MgCl_2_ 1.0 mmol/L, CaCl_2_ 1.8 mmol/L) and incubated with Bocillin 10, 50 or 100 ug/ml for 10 or 30 minutes. After incubation the cells were washed in HBSS buffer and observed by fluorescence inverted microscopy (Leica Microsystems GmbH, Germany).

To confirm the cellular uptake of Penicillin, we performed a flow cytometry analysis. After trypsinization, podocytes (5×10^5^ cells/ml) were incubated with 10 ug/ml Bocillin for 20 minutes. Cells were washed with cool PBS and resuspended in Penicillin-free medium. At the indicated times 1.5×10^3^ cells were analyzed by flow cytometry (Bekton Dickinson FACS Elite) and untreated podocytes were used as control.

### MTT assay

Human immortalized podocyte proliferation was assessed by the methylthiazoletetrazolium (MTT) assay (Sigma Company, St. Louis, MO, USA), according to the manufacturer’s instructions. This non-radioactive cell proliferation assay identifies living cells based on the cellular conversion of a tetrazolium salt into a formazan product, a chromaphore which can be quantified by ELISA. Briefly, cells were plated onto 96 multi-well plates (8000 cells/well) and allowed to adhere overnight without antibiotic. Podocytes were exposed to PA alone (10, 5 and 2.5 ug/ml), Penicillin G alone (10, 50, 500 and 700 Units/ml) or PA and Penicillin G at the same concentration, in medium containing 1% fetal bovine serum (FBS). After 48 h the medium was removed and cells incubated with fresh medium containing MTT (0.5 mg/ml) for 3 hours. After removing the MTT-containing medium, 200 ul of dimethylsulfoxide (DMSO) was added and the plates were immediately read at 570 nm. Wells containing no cells (but containing medium and MTT over the incubation period) were used to blank the plate reader. The results were the means of three separate experiments, expressed as absorbance at 570 nm.

### Transporter gene expression study

Gene expression of various Penicillin G membrane transporters, selected according to the data reported for other cell types, were analyzed in human and rat podocytes. Specifically, we investigated organic anion transporters of the OATP family, one transporter of the OAT family, the peptide transporters PEPT1 and PEPT2, and the efflux transporter P-glycoprotein. As a control, the same transporters were analyzed in neuronal (SH-SY5Y neuroblastoma) and intestinal cell lines (Caco2 colon cancer cells), as well as in whole organ mRNA extracts (intestine, liver, and kidney).

Total RNA from cells was extracted using the Invitrogen Pure Link TM Micro-to-midi Total RNA Purification System. RNA concentrations were determined using Nanodrop ND 1000 (Cell Euroclone Italy). One microgram of total RNA was reverse transcribed using MMLV reverse transcriptase (Applied Biosystems). The analyses were performed by transcriptase-polymerase chain reaction (RT-PCR) and quantitative Real Time RT-PCR (QRT-PCR). Primers and annealing temperatures are reported in Table 2 and Table 3; GAPDH and beta-actin were used as house-keeping genes, as appropriate.

**Table 2:** Investigated human transporters.

Type PCR	*GBN*	*Protein and Gene Symbol*	*Primer pair*	*TA (°C)^a^*	*Amplif. region*	*Length(bp)*
RT-PCR/QRT-PCR	NM 134431	OATP1A2, (*SLCO1A2)* OATP-A	(F) *5’*-CCATTGGAACGGGAATAAACA-*3’* (R) *5’*-TCTCTTCAGATTTCATACACCTCA -*3’*	60°	2136–2351	216
	NM 007256	OATP2B1, (*SLCO2B1)* OATP-B	(F) *5’*-GGACAACAGCCAGGTTTTCTACAC-*3’* (R) *5’*-AGGAAGGGCACCACCAGATG-*3’*	60°	1851–1958	108
	NM 006446	OATP1B1, (*SLCO1B*1) OATP-C	(F) *5’*-TAAGGCTAACATCTTATTGGGAGTC-*3’*(R) *5’*-ACAGCAGTAAAACATGAGAATTTGG-*3’*	60°	1250–1382	133
	NM 013272	OATP3A1, (*SLCO3A1)* OATP-D	(F) *5’*-AGCCCTGGACCCCTACTCG-*3’*(R) *5’*- CCCGTGAGATTCGTGCTGTTG-*3’*	60°	1582–1716	135
	NM 016354	OATP4A1, (*SCL21A12)* OATP-E	(F) *5’*-CACCAGTTGAAGGACAGCAG-*3’*(R) *5’*-AGGAGCCAGATGGAGAGAGG-*3’*	60°	1253–1341	89
	NM 004254	OAT3 (*SLC22A8*)	(F) *5’*-CCCACAGTCATCAGGCAAACA-*3’*(R) *5’*-AGGGCGGTGATCCCGTAGA-*3’*	60°	1448–1584	137
	NM 000927	MDR1 *(ABCB1)*	(F) *5’*- TGCTCAGACAGGATGTGAGTTG-*3’*(R) *5’*-AATTACAGCAAGCCTGGAACC-*3’*	60°	2808-2926	122
	NM 005073	PEPT1 (SLC15A1)	(F) *5’*- CACCTCCTTGAAGAAGATGGCA-*3’*(R) *5’*- GGGAAGACTGGAAGAGTTTTATCG-*3’*	60°	1121-1225	105
	NM 021082	PEPT2 (SLC15A2)	(F) *5*’-TTTGTCTCTCTACACTGAGCATTC-*3′*(R) *5′* -CTGCTTTCTGTATCCTTTACCATC-*3′*	60°	1453-1563	111
	NM 002046	GAPDH	(F) *5′-*CCCATCACCATCTTCCAGGAG*-3′*(R) *5′-* CTTCTCCATGGTGGTGAAGACG*-3′*	60°	319-423	105
Only RT-PCR	NM 005073	PEPT1 (*SLC15A1)*	(F) *5′*-TCAGGTCGGAGGAGTAGC-*3′*(R) *5′* -AGAATTGGCGTCAGGTAGC-*3′*	55°	4-283	279
	NM 021082	PEPT2 *(SLC15A2)*	(F) *5′*- GAAGCCATCTCCGACAATCTG-*3′*(R) *5′* -GCCAAGCACATACACCAAGG -*3′*	60°	245- 525	280

GBN Gene Barnk Number; TA Annealing Temperature.

**Table 3:** Investigated rat transporters.

Type PCR	GNB	*Protein and Gene Symbol*	*Primer pair*	*TA (°C)*	*Amplif. region*	*Length (bp)*
RT-PCR	AF257746.1	Mdr1a (abcb1a)	(F) *5′-*GGGCACATGATCAAGACGGGG*-3′*(R) *5′-* GAGCAGCGTCAT TGGCAAGCCTGG*-3′*	65°	2081-2531	450
	NM 012623.2	Mdr1b(abcb1b)	(F) *5′-*AGTGACACTGGTGCCTCTGA*-3′*(R) *5′-* CAAACACTGGTTGTATGCAC*-3′*	62°	1965-2210	245
	D50664.1	PepT1 (Slc15a1)	(F) *5′-* GCACCCTTAACGAGATGATCACC*-3′*(R) *5′-* AGGCGAACAGAACATACTCAGG*-3′*	60°	1529-2018	489
	NM 031672.1	PepT2 (Slc15a2)	(F) *5′-* GAGTATCTCCAGCATGCTGGTCAAGG*-3′*(R)*5′-*CCCAACTGCAACGGTCAACAACCAGGCC*-3′*	62°	1667-2147	480
	AB17446.1	Oat3 (Slc22a8)	(F) *5′-* CATCTTGCCTGGTGCCATGAC*-3′*(R) *5′-* TACTGCTTGGGATCAGTCTCTTGTG*-3′*	55°	108-1792	1684
	NM 030838.1	Oatp3 (Slco1a5)	(F) *5′*-CGCTTGGGATTGGATTACATGC-*3′*(R) *5′* -ATGAGACAGTGGGGTTTGGAGA-*3′*	57°	1870-2482	612
	NM 1336082	OatpE (Slco4a1)	(F) *5′*- CAGGTTGAGAAACGGAGCAG-*3′*(R) *5′* - GATGGCAATATAGATGGGCG-*3′*	57°	181-816	635
	NM 031144	beta-actin	(F) *5′-*GACGACATGGAGAAGATCTGG*-3′*(R) *5′-* GAGGATGCGGCAGTGGCCAT*-3′*	58°	298-790	492
QRT-PCR	NM 017111.1	Oatp1 (Oatp1a1)	(F) *5′*-CTGCCTGCCTTCTTCATTCTGA-*3′*(R) *5′* -GCTTTCCTTCTCTCCGGGCATC-*3′*	55°	1897-2000	103
	U95011	Oatp2 (Oatp1a4)	(F) *5′*-TGGCATTCCTGCACCCATT-*3′*(R) *5′* -TGTCATACATCCTGCATGCCC-*3′*	55°	1891- 1995	104
	NM 1336082	OatpE (Slco4a1)	(F) 5-CTGGTTCTCGTGTTCGTTGTAATT-3(R) 5-CACAGACACATCGTAGAGTAGCAGTTAG-3	60°	1874-1926	52
	NM 001002024.1	Oatp4c1	(F) *5′*-GCAAGGTATTGTAGTAAATGGCCTAGT-*3′*(R) *5′* - AGACAACACGCAAAAGGAGATGT-*3′*	58°	338-465	127
	AY5825225	Mdr1a (accb1a)	(F) *5′*-ATCAACTCGCAAAAGCATCC-*3′*(R) *5′* -AATTCAACTTCAGGATCCGC-*3′*	60°	1973-2089	116
	BC107560	Mdr1b (abcb1b)	(F) *5′*-TCGTTGCCTACATCCAGGTT-*3′*(R) *5′* -CAGCGTCATTCACGT CAAAC-*3′*	53°	508-634	*126*
	X02231.1	GAPDH	(F) *5′*-TAAAGGGCATCCTGGGCTACACT-*3′*(R) *5′* -TTACTCCTTGGAGGCCATGTAGG-*3′*	60°	873-1073	200

GBN, Gene Barnk Number; TA, Annealing Temperature;

For the QRT-PCR the amplification steps were: pre-denaturation at 95°C for 10 min, 40 cycles of amplification with denaturation at 95°C for 15 s, annealing at proper temperature for 60s and extension at 72°C for 30 s. A final extension at 72°C for 10 min and a dissociation stage (95/60/95°C for 15 s each) were then added.

RT-PCR conditions were described by Tramonti et al. [1] and Engel et al. [14]. For the RT-PCR the ethidium bromide-stained agarose gel was visualized using a gel documentation system (PhotoDoc-it, Imaging System Digital, UVO Cambridge UK).

### Transporter immunofluorescence analysis

An indirect immunofluorescence method was utilized on primary cells fixed in acetone or paraformaldehyde, depending on the subsequent application, and plated on Thermanox plastic coverslips (Nunc, Rochester, NY, USA). F-actin was detected directly by phalloidin-FITC or phalloidin-rhodamine (Sigma). Mouse monoclonal anti-[C219] P-glycoprotein (Abcam), rabbit anti-synaptopodin and rabbit anti-vinculin (Sigma) were the primary antibodies used for the study. As secondary fluorescent-labelled antibodies, we used FITC-conjugated goat anti-mouse IgG (Pierce), FITC-conjugated goat anti-rabbit IgG (DAKO A/S, Nenmark) and Alexa Fluor 488 donkey anti-rabbit (Invitrogen). Slides were examined by a fluorescence microscope (Leica Microsystem, Germany). Controls with no primary antibody showed no fluorescence labelling. P-glycoprotein expression was analyzed semi-quantitatively measuring fluorescence intensity by image analysis software (Image ProPlus 6.3 Software, Media-Cybernetics, SilverSpring, MD, USA). Results were expressed as relative intensity comparing treated cells to controls. For each experimental point, 10 to 20 microscopic fields were examined.

### Flow Cytometry Analysis of P-glycoprotein activity

P-glycoprotein-related transport activities were investigated by using the fluorescence probe Rho123 (Sigma Company, St. Louis, USA) in an efflux assay, as described by Chen et al. [15]. After PA incubation for 48 hours, human podocytes were tested for Rho123 efflux rate. Podocytes (5×10^5^ cells/ml) were washed and stained with 200 ng/ml Rho123 for 20 minutes. Cells were washed again with cool PBS and resuspended in Rho123-free medium for 60 min at 37°C to allow for Rho 123 efflux. At the indicated times 1.5×10^3^ cells were taken for analysis on a flow cytometer (Beckton Dickinson FACS Elite). Podocytes not treated with Rho123 were used as control. Cyclosporine A (CSA 0.1, 0.5 or 1 uM) was used to inhibit P-glycoprotein activity and added to the Rho123-free medium after staining to prevent probe efflux. A minimum of 15,000 gated events were recorded for each sample.

### Membrane transporters’ blockade

As transport inhibitors we used cyclosporine A and rifampicin (Sigma Company, St Louis, UAS). While rifampicin blocks the OATPs/Oatps transporters, cyclosporine A exerts its inhibiting activity on both OATPs/Oatps and P-glycoprotein. The two inhibitors were alternatively utilized in combination with fluorescent penicillin. More in detail, to assess effects on OATPs/Oatps activity, cells were first treated for 30 minutes with Cyclosporine 1 uM, or rifampicin 1 uM–10 uM. Then, fluorescence penicillin (50 ug/ml) was added for 30 minutes; after washes, live cells were imaged.

To study P-glycoprotein blockade, cells were first incubated with fluorescent penicillin 50 ug/ml for 30 min, and images were taken after addition of cyclosporine 1 uM for 30 min.

Fluorescence intensity was measured on 100 cells per condition by image analysis software (Image ProPlus 6.3 Software) and results were expressed as relative change of intensity compared to controls arbitrarily given a value of 1. Experiments were repeated trice per each condition.

### Statistical analysis

Data are presented as mean ± SD or mean ± SEM. Comparison of means was performed by ANOVA test.

## Results

### Penicillin G pre-treatment in isolated glomeruli before PA incubation

PA incubation at concentrations ranging from 10 ug/ml to 0.6 ug/ml increased P_alb_ of isolated healthy glomeruli (Fig 1a). The effect was abolished in a dose-dependent manner by 15 min pre-incubation with Penicillin G and complete inhibition appeared at a concentration of 700 IU/ml, but a significant effect was already present at a concentration of 500 IU/ml (Fig. 1b).

**Figure 1:** Albumin permeability (Palb) assay in isolated glomeruli from healthy rats. (a) Palb increases after PA incubation (***P<0.0001 vs NT - untreated glomeruli), and the increase is completely blocked (b) by preincubation with Penicillin G (PEN), when 700 Units/ml are added to the cells and is reduced by 500 Units/ml (**P<0.001, ^***^ *P*<0.0001 and ^#^ *P*<0.05 vs. corresponding PA concentration). (c) The incubation with Penicillin G alone does not alter glomerular albumin permeability, and (d) treatment with Penicillin G after PA incubation does not protect glomerular integrity (*** *P*<0.0001 vs NT). P_alb_ values are expressed as mean ± standard deviation. 25 glomeruli were analyzed per each point.

Incubation of glomeruli with Penicillin G alone did not affect P_alb_ (Fig. 1c). When isolated glomeruli were exposed to PA (10 ug/ml) before Penicillin (700 Unit/ml), P_alb_ remained elevated (0.75±0.05 vs. 0.89±0.20) (Fig. 1d), supporting the hypothesis that the Penicillin effect is exerted by blocking PA entrance into the cell.

### Effect of PA and Penicillin G on glomerular adhesion and cellular outgrowth on collagen IV substrate

In control conditions 85±5% of isolated glomeruli adhered to the collagen IV substrate, and a cellular outgrowth was observed around the glomerular structure (Fig. 2A-a). The incubation with PA alone diminished the number of adhered glomeruli at all PA concentrations compared to control; the outgrowth from glomeruli was limited, and the cellular morphology was altered (Fig. 2A-b, 2B).

**Figure 2:** Glomerular adhesion and cellular outgrowth. A. The images show glomerular adhesion and cellular outgrowth in: (a) control conditions, (b) after addition of PA 2.5 ug/ml, and (c) when Penicillin G (700 Units/ml) is added before PA treatment. B. The graph represents the percentage of adhered glomeruli compared to untreated controls; isolated glomeruli were pre-incubated with PA alone (10, 5 and 2.5 ug/ml), or Penicillin G (500–700 Units/ml) followed by PA. The percentage of adhered glomeruli increases with Penicillin G pre-treatment, albeit reaching statistical significance only for Penicillin G 700 Units + PA 2.5 and 5 ug/ml. Scale bars  =  100 um.^ #^ *P*<0.05 ^**^ *P*<0.001 vs. PA-treated glomeruli.

A complete inhibition of the PA effect was present when Penicillin G 700 IU/ml was pre-added, i.e. the number of attached glomeruli and the outgrowth from glomeruli were similar to the control experiment (Fig. 2A-c, 2B). A partial inhibition of PA effect was observed for Penicillin G 500 IU/ml (Fig 2B). Glomeruli treated only with Penicillin at the same concentrations demonstrated a behavior similar to the control (data not shown).

### Penicillin G prevents PA-induced podocyte damage

A preliminary time-course study was first conducted with human podocytes incubated with PA for different periods (12, 24, 32 and 48 hours); decreased viability was observed after 48 hours of incubation; therefore, this time point was selected for further investigation.

Penicillin G alone did not affect cell viability as compared to medium alone, whereas PA alone diminished viability by about 50% (Fig 3a). Pre-incubation with Penicillin G prevented partially or completely the decrease of viable cells induced by PA; the effect was statistically significant at the concentration of 700 IU/ml of Penicillin G (Fig 3a).

**Figure 3:** Cell viability and cytoskeleton organization. (a) MTT assay results: Penicillin G alone does not affect podocyte viability at any used concentration from 50 to 700 IU/ml (group bars on the left). PA-induced loss of viability (black bars) is not influenced by pre-incubation with 50 IU/ml penicillin (light rose bars), whereas it is dose-dependently prevented by 100, 500 and 700 IU/ml Penicillin G (dark violet, light violet and gray bars). Best effects of Penicillin are observed at lower doses of PA (2.5 ug/ml, group bars on the left). Graph bars indicate mean ± SD values from three independent experiments. **  =  *P*<0.001 vs. PA alone, ^#^ *=  P*<0.05 vs PA alone. (b) Double staining for vinculin and actin. In control condition, vinculin is periodically expressed at the cell periphery, at the tip of actin stress fibers, as shown by co-localization with actin (left panels). These features are modified after incubation with either 2.5 and 10 ug/ml PA; vinculin is irregularly dispersed in the cell body, actin stress fibers are progressively reduced by 2.5 and 10 ug/ml PA, and co-localization of the two molecules occurs in the cell body and is absent at the cell periphery (middle panels). Preincubation with Penicillin G (500 Units/ml) partially (PA 10 ug/ml) or completely (PA 2.5 ug/ml) preserves the cytoskeletal structure from PA damage (right panels); the antibiotic prevents loss of actin fibers even with PA dosages of 10 ug/ml. With 2.5 ug/ml PA, vinculin-positive focal adhesions are also maintained at their location. Scale bars  =  20 um.

As illustrated in Figure 3B, in control condition actin stress fibers were prominent in the podocyte cell body. The focal adhesion molecule vinculin showed a peripheral and regularly distributed pattern of expression and co-localized with actin. These features were dose-dependently lost after PA incubation (2,5 and 10 ug/ml) for 48h, whereas preincubation with Penicillin G partially (PA 10 ug/ml) or completely (PA 2.5 ug/ml) prevented PA-induced cytoskeletal remodeling.

### Internalization of fluorescent Penicillin in human podocytes

The above described results suggest that Penicillin G may block PA entry by engaging membrane transporters. If so, it would be possible to find Penicillin G inside the cell. To test this hypothesis, cells were incubated with the Penicillin fluorescent analogue Bocillin. Fluorescent intracellular puncta evenly distributed throughout the cytoplasm (Fig. 4a,b,c) and in the cell processes (Fig 4d, e) were clearly observed after 30 minutes incubation. Intracellular fluorescence was detected in 100% of cells also by flow cytometry (Fig 4f).

**Figure 4:** Internalization of fluorescent Penicillin. (a, b) After 30 min incubation with the fluorescent Penicillin G analogue, intracellular fluorescence is clearly observable in the cell body as well as in the cell processes, as better detailed in (d). Panel c) is the corresponding brightfield image of (d). Panel e) is the negative control. Panel f) displays the results obtained by evaluating cell fluorescence by flow cytometry and shows that all cells (99.9%) were fluorescent (blank histogram  =  autofluorescence region (AU); gray histogram  =  intracellular fluorescence. Scale bars  =  10 um.

### Penicillin G pre-treatment in the PA rat model

As expected [16], a single injection of PA in three-month old Sprague-Dawley rats caused proteinuria by day 10 (52.41±19.51 vs. 9.86±2.87 mg/d), soon accompanied by decreased serum albumin (1.68±0.26 vs. 3.12±0.45 g/dl, Table 4). Pretreatment with either 12,500 or 15,000 IU Penicillin G reduced proteinuria (14.18±8.3 and 15.14±12.25 vs. 52.41±19.51 mg/d), and was associated with increased serum albumin (Table 4). Penicillin pre-treatment also affected the kidney-to-body weight ratio and glomerular size. Control animals, receiving Penicillin G followed by saline, did not differ from saline-injected controls (Table 4). The analysis of P_alb_ on isolated glomeruli from animals sacrificed at the end of the study (day 10) showed that Penicillin G pre-treatment preserved glomerular albumin permeability in the normal range and demonstrated a strict correlation with the urinary protein values observed in the in vivo experiments (Fig 5).

**Table 4:** Variables (mean ± standard deviation) at the end of the animal study.

Analysis	Control 1	Experimental 1	Experimental 2	Experimental 3	Control 2	Control 3
Proteinuria (mg/24h)	9.86±2.87	2.41±19.51^#^	14.18±8.3	15.14±12.25	12.83±8.04	13.75±5.05
Serum albumin (g/dl)	3.12±0.45	1.68±0.26^**^	2.23±0.95	2.73±0.68	3.35±0.27	3.23±0.25
Serum creatinine (mg/dl)	0.25±0.02	0.37±0.13	0.32±0.02	0.29±0.64	0.26±0.03	0.28±0.15
Renal weight (mg/g body weight)	3.02±0.13	5.08±1.21^**^	3.16±0.10	3.93±0.95	3.25±0.11	3.61±0.27
Glomerular area (µm^2^×10^3^)	7.8±0.5	10.6±1.7^**^	8.8±0.7	8.3±0.7	7.05±1.02	7.36±0.80
Glomerular permeability (P_alb_)	0.03±0.03	0.71±0.13^**^	0.16±0.24	0.07±0.23	0.07±0.26	0.02±0.14

Control 1, saline; Control 2, PEN 12,500; Contro 3, PEN 15,000; Experimental 1, PA; Experimental 2, PEN(12,500)+ PA, Experimental 3, PEN (15,000)+ PA.

PA, puromycin aminonucleoside; PEN Penicillin G; **^#^** *P*<0.005 compared with control 1;** *P*<0.05 compared with control 1 ;^ **^ *P*<0.0001 compared with control 1.

**Figure 5:** PA rat model. Panel a) shows the results of Palb values in glomeruli isolated from rats treated with PA compared to controls and Penicillin-injected animals. P_alb_ values are expressed as mean ± SD, and 25 glomeruli were evaluated per each animal (5 rats per group). ^###^ *P*<0.00001 vs. controls **P<0.001 vs. PA model *** *P*<0.0001 vs. PA model. Panel b) displays the urinary protein determination obtained from the same groups of rats. Values are expressed as mean ± SD. ^# #^ *P*<0.005 vs. controls.

### Podocytes express the mRNA of species-specific membrane transporters

The inhibitory effect of Penicillin G on PA-induced glomerular injury both in vitro and in vivo, and the entrance of Penicillin into the cell, suggested the possible engagement by Penicillin of the same membrane transporters used by PA. Therefore, RT-PCR and quantitative RT-PCR experiments were performed to analyze components of the membrane transport families that have been associated with Penicillin G membrane transport in other cell systems.

As summarized in Fig 6, human podocytes expressed OATP-A, OATP-B, OATP-D and OATP-E from the OATP family; in contrast, OATP-C (liver specific transporters), OAT3 and PEPT1 were not detected, and PEPT2 showed a low expression level (Fig 6a, b). In primary rat podocytes, we studied the OATP transporter family (Oatp1, Oatp2, Oatp3, OatpE, Oatp4c1), one member of the Oat family (Oat3), and the peptide transporters PepT1 and PepT2 (Fig 6c,d). In agreement with the results obtained in human cells, we found expression of all genes that codify for Oatp transporters but Oatp3, and absence of the other analyzed membrane transporters.

**Figure 6:** Transporter gene expression in human and rat podocytes. Results from RT-PCR and QRT-PCR analysis of membrane transporters in human cell lines (a,b) and primary rat podocytes (c,d). (a) RT-PCR analysis of human cells lines; P  =  human podocytes, N SHSY-5Y =  neuroblastoma cells; I Caco2  =  colon cancer cells. (b) QRT-PCR analysis of membrane transporters using the same primers in human podocytes. (c) RT-PCR analysis of primary rat podocytes; the results compare gene expression of cells obtained from three distinct isolation procedures (I, II, III). (d) QRT-PCR analysis of Oatps members in primary rat podocytes. Results are expressed as mean ± SEM of three independent experiments. NTC  =  RT-PCR negative control.

Considering the high expression of the OATP transporters, we searched for their possible variation induced by PA. Though a significant variation was only found for Oatp2, that was increased in rat podocytes after PA treatment, also other transporters exhibited expression changes, particularly OATP-A in human cells and Oatp1 in rat podocytes (Fig 7a,b,c).

**Figure 7:** Membrane transporter analysis after PA treatment in human and rat podocytes. QRT-PCR analysis of membrane transporters in the human podocyte line (a,b) and primary rat podocytes (c); human podocyte gene expression was evaluated at 24 (a) and 48 hours (b) after PA treatment; (c) primary rat podocytes were evaluated after 48 hours. Results are expressed as mean ± SEM of three independent experiments. ^#^ *P*<0.05.

### Podocytes express a specific efflux transporter P-glycoprotein

The gene expression of OATP/Oatp influx transporters on the podocyte surface implies the co-expression of efflux membrane transporters, such as P-glycoprotein, as described by Kim [17].

Our results show that the P-glycoprotein transporter gene (MDR1) is indeed expressed by human podocytes (Fig 8a), and increases in PA-treated cells, particularly after 48 hours (P<0.001, Fig 8c).

**Figure 8:** Gene expression analysis of P-glycoprotein in human and rat podocytes. (a) PCR analysis of MDR1 in human podocytes. (b) PCR analysis of Mdr1a and Mdr1b in rat podocytes. NTC  =  RT-PCR negative control. Panel (c) shows the increase of MDR1 after 24 and 48 hours of PA incubation in human podocytes, and panel (d) displays the variation in Mdr1a and Mdr1b expression in rat podocytes. Results are expressed as mean ± SEM of three independent experiments. ^#^ *P*<0.05 ^* *^ *P*<0.001.

Correspondingly, the rat MDR1 homologues, Mdr1a and Mdr1b, are both expressed in rat podocytes (Fig 8b), where 48 hour PA incubation was able to increase Mdr1a expression (Fig 8d).

P-glycoprotein analysis by immunofluorescence confirmed the increased expression after 48 hour PA incubation (Fig 9 a,b,c), when PA also caused remodeling of the podocyte cytoskeleton, as shown by the alteration of synaptopodin (Fig 9e), and the almost complete disappearance of actin stress fibers (Fig 9g).

**Figure 9:** P-glycoprotein expression and cytoskeletal organization in primary rat podocytes. Compared to cells maintained in control conditions (a), PA-treated (10 ug/ml for 48 hours) primary podocytes show increased expression of P-glycoprotein, which is evident by immunostaining (b) and appears significant by semi-quantitative analysis of immunofluorescence (c) (^***^ *P* <0.0001 compared to NT). PA-treated cells also display reduced synaptopodin (e) and actin expression (g) as compared to untreated cells (d,f). Scale bars  =  50 um.

To establish if P-glycoprotein expressed by podocytes was functionally active, and if its activity could be modified by PA, we used its specific fluorescent substrate Rho 123 (Fig 10) and the specific inhibitor cyclosporine A (CSA) [15]. In control experiments, after Rho 123 incubation and replacement with Rho 123-free medium, mean fluorescence intensity decreased by approximately 35%, indicating Rho 123 efflux from the cells (Fig 10a). PA incubation caused an increase of Rho 123 efflux, as shown by further reduction of fluorescence as compared to the control cells (Fig. 10b), whereas CSA consistently abolished the efflux of the substrate.

**Figure 10:** P-glycoprotein activity. Panel (a) shows representative histograms of Rho 123 fluorescence variation in the human podocyte cell line after PA (10 ug/ml) or cyclosporine A (CSA) (1 uM) treatment for 48 hours or incubation with medium alone (NT). The white area in the right upper panel corresponds to the autofluorescence region (AU). The values (P) in the figure indicate the percentage of fluorescent cells. Panels b) and c) illustrate PA and CSA effects on Rho 123 exit from the cells. Results are expressed as mean ± SD of three independent experiments. ^#^ P<0.05 vs NT, ^***^ *P*<0.0001 vs.NT.

### Effects of transport blockade

Confirming the use of OATPs/Oatps by penicillin G to enter the cell, blockade of these transporters by either cyclosporine or rifampicin, inhibited the entry of fluorescent penicillin (Figure 11a,b) into podocytes.

**Figure 11:** OATPs and P-glycoprotein blockade. a) Inhibition of OATPs by cyclosporine. Incubation of cells with vehicle (30 min), followed by fluorescent penicillin (30 min) (NT) results in a diffuse cytoplasm fluorescent signal indicating that penicillin has entered the cell (left panel). If cyclosporine (CYCLO) is added before penicillin (right panel), most cells are negative, indicating the blockade of influx transporters (^***^ *P*<0.0001 vs NT). b) Inhibition of OATPs by rifampicin. The left image represents an example of control cells incubated with vehicle followed by penicillin, showing entrance of the antibiotic as witnessed by fluorescent cytoplasm signal. On the right, 10 uM rifampicin is able to inhibit the entry of penicillin, and cells do not contain fluorescent material (^**^ *P*<0.001). c) P-glycoprotein blockade by cyclosporine. The left image shows representative cells incubated with fluorescent penicillin for 30 min, followed by vehicle for additional 30 min. At this time point, penicillin has almost completely left the cells, which are mostly negative by immunofluorescence. On the right, the image shows cells incubated with fluorescent penicillin for 30 min, followed by cyclosporine for additional 30 min. Retention of fluorescence indicates the blockade of efflux transporters by cyclosporine (^##^ *P*<0.005). Graphs show the results of digital measurement of fluorescent intensity, obtained from three different experiments and on 100 cells/experiment. Results are expressed as mean ± SEM. Bar = 50 um.

When cyclosporine was added after penicillin internalization was completed, P-glycoprotein blockade was confirmed by persistent cell fluorescence, whereas untreated cells were mostly devoid of penicillin (Figure 11c).

## Discussion

The presence of aminoacid transporters in podocytes has been known for some time [4], whereas drug transport has been largely investigated only in tubular cells [5]. As a basis for the present experiments, we speculated that substances which are harmful to the podocyte, such as Puromycin Aminonucleoside (PA), require a drug transporter system to enter and damage the cell.

The membrane transporters OATLP1 and mOCTL1 have been described in podocytes, and have been shown to contribute to trans-epithelial molecular transfer in these cells [2], [3]. More recently, Xia e al. [6] suggested that PA uses a membrane transporter to enter the podocyte, and our expression data demonstrate that, besides the organic cation transporter PMAT identified by these authors, podocytes do express and utilize other transporters for which Penicillin G is a known substrate. Further support to our results comes from a series of microarray expression data obtained from mouse primary podocytes or mouse podocyte cell lines, publicly available as GEO data sets (for instance: GSM253173, GSM253174, and GSM833242, GSE17145, and GSE39441). They show that podocytes indeed express a complete series of drug transporters of the OATP and MDR families, as well as of the OAT/OCT family.

The potent Penicillin G prevention of PA-induced increased glomerular permeability and of the accompanying harmful consequences on podocyte cytoskeletal structure can only be explained by the sharing of the same transport systems by the two substances. In line with this hypothesis, fluorescent Penicillin was observed inside the cell, while administration of Penicillin after PA was ineffective, still consistent with a cis-inhibition of the uptake mechanisms.

Drug transporter molecules have been classified into influx transporters, related to the uptake of substances into the cell, and efflux transporters, which are involved in the transport of materials outside the cell, and are typically located either at the basolateral or the apical membrane in polarized cells [17].

The OATP transporters have been considered key determinants in the cellular uptake of many endogenous and exogenous chemicals and are expressed in various tissues [17], [18]. They were long considered only transporters of organic anions, but have also been shown capable of transporting cation, neutral, zwitterionic as well as anionic compounds [17]. Recently, the OATP family has been identified as the main transporter of Penicillin G in humans [19].

The proton-coupled oligopeptide transporters PEPT1 and PEPT2 have a significant role in conservation and regulation of peptide-bound amino acids and also in the absorption, availability and efficacy of a variety of peptidomimetic drugs, such β-lactam antibiotics [1].

Our results show that the mRNA of components of the OATP/Oatp families, and at a much lesser extent those of the PEPT family, are expressed by both human and rat podocytes. Expression of OATP members is affected by PA treatment, both in vitro and in vivo. In contrast to podocytes, renal tubular cells handle Penicillin G mainly by the OAT3 transporter, and accordingly, Oat3 knockout mice exhibit altered clearance and distribution of the antibiotic [20]. An exact homology between OATP transporters in humans and Oatp transporters in rodents does not exist, and several components of this transport family are still unknown. Rat Oatp1 and Oatp2 are abundantly expressed in liver and kidney and much less in the brain, whereas Oatp3 is absent in the liver but highly expressed in the kidney [21]. According to our data, podocytes seem to express both Oatp1 and Oatp2, but not Oatp3. Human OATPE and rat OatpE have an overall aminoacid sequence homology of 72.6% and have been found in the retina [22]. In contrast, the expression of Oatp4c1 was described specifically in rat glomeruli [23], in agreement with our data.

Concerning the efflux transporters, Kim et al. [17] showed that a number of OATP transporters share drug substrates with certain efflux transporters, such as P-glycoprotein (MDR1), and this co-expression is described in several organs involved in drug disposition such as the liver, the intestine, and kidney tubular cells, as well as in barrier systems, such as the blood brain barrier. P-glycoprotein acts as a membrane-bound, ATP-consuming drug efflux pump that actively extrudes a variety of structurally unrelated compounds across the plasma membrane as a defense mechanism [1]. Thus, the coordinated activity between an OATP influx transporter and an efflux transporter may determine the net cellular drug entry or efflux of shared substrates [17]. Functionally, two different types of P-glycoprotein have been described, but only class I has been related to drug transport [24]. Humans carry a single class I group gene (MDR1, or ABCB1 ATP-binding cassette, sub-family B (MDR/TAP), member 1), while rodents carry two class I genes (mdr1a and mdr1b) (1); all encoded proteins are capable of drug transport, and Penicillin G is their main substrate [25].

We discovered a significant expression of the genes encoding P-glycoprotein in human and rat podocytes, and, similarly to OATP/Oatp molecules, their expression changed after PA treatment. In vitro, we could also confirm increased extrusion activity after PA treatment, which could be an important mechanism of protection from pathological insults, albeit not podocyte-specific, because mesangial cells have been shown to possess this protein as well [25].

Our studies with specific inhibitors of confirm that both influx and efflux transporters are actively engaged by Penicillin G on the podocyte surface. Therefore, based on results obtained in this study, we can summarize our working hypothesis as represented in Figure 12; podocytes constitutively express specific membrane transporters which regulate small solute passage across the membrane and maintain cellular homeostasis. For example, low dosages of Penicillin G are dealt by these transporters and podocytes do not exhibit morphological and molecular changes. Due to its chemical characteristics, PA uses the same membrane transporters as Penicillin G to enter podocytes, but PA entry causes podocyte damage and variation of expression of the transporters themselves. Instead, when membrane transporters are already engaged by Penicillin G, PA entry is blocked and cell damage is prevented.

**Figure 12:** Proposed working model. a) In physiological conditions, influx and efflux transporters deal with small solutes and contribute to the maintenance of podocyte structure. b) Low doses of Penicillin G use influx and efflux transporters and do not cause podocyte damage. c) Entrance of PA causes podocyte damage. In addition, cells incubated with PA display changes of expression of transporters, especially intense for efflux molecules. d) Engagement of influx transporters by Penicillin prevents the entrance of PA, that cannot exert its damaging effects on the cell.

In conclusion, our study has demonstrated the existence and function of some influx and efflux membrane drug transporters on podocytes and their modification in response to PA. Further research is certainly needed to completely clarify their function, which could be relevant for cell pathophysiology and the choice of treatment for glomerular diseases. Considering that membrane transporters are involved in drug metabolism, we believe that specific polymorphisms of these molecules may be relevant to drug response in nephrotic syndrome.
